The article "The Safety and Efficacy of Standard-Dose versus Low-Dose Non-Vitamin K Antagonist Oral Anticoagulants in Patients with Nonvalvular Atrial Fibrillation and Left Atrial Appendage Thrombus" was published in 2021. Journal: J Healthc Eng.

# The Safety and Efficacy of Standard-Dose versus Low-Dose Non-Vitamin K Antagonist Oral Anticoagulants in Patients with Nonvalvular Atrial Fibrillation and Left Atrial Appendage Thrombus

**DOI:** 10.1155/2021/1839399

**Published:** 2021-12-15

**Authors:** Mingjun Feng, Huaming Lin, Bin He, Binhao Wang, Xiaomin Chen, Huimin Chu

**Affiliations:** ^1^Arrhythmia Center, Ningbo First Hospital, Ningbo 315000, China; ^2^Department of Cardiology, Quhua Hospital, Quzhou 324000, China

## Abstract

**Background:**

Data comparing different doses of non-vitamin K antagonist oral anticoagulants (NOACs) regarding resolution of left atrial appendage thrombus (LAAT) in patients with nonvalvular atrial fibrillation (AF) are scarce. This study aimed to investigate the safety and efficacy of standard-dose versus low-dose NOACs in patients with nonvalvular AF and LAAT.

**Methods:**

Patients with nonvalvular AF who underwent transesophageal echocardiography (TEE) before interventional procedures for the detection of LAAT and treated with NOACs from October 2014 to September 2020 in Ningbo First Hospital were retrospectively screened. The study population was divided into two groups according to the doses of NOACs: standard-dose group (dabigatran 150 mg, twice daily; rivaroxaban 20 mg, once daily) and low-dose group (aged ≥75 years, body weight <50 kg, or creatinine clearance <50 mL/min; dabigatran 110 mg, twice daily; rivaroxaban 15 mg, once daily). Repeated TEE was performed 1, 2, and 3 months later. The rate of LAAT completely resolved and incidence of thromboembolic and major bleeding events were compared between the two groups.

**Results:**

A total of 24 patients were included, 14 patients in the standard-dose group and 10 in the low-dose group. After 3 months, LAAT was completely resolved in 12 out of 14 (85.7%) and 8 out of 10 (80%) patients treated with standard- and low-dose NOACs, respectively. The rate of LAAT completely resolved was comparable between groups. No thromboembolic or major bleeding events occurred during the follow-up.

**Conclusion:**

Low-dose NOACs are a safe and effective option for the treatment of LAAT in some special subset patients. However, the results warrant validation in a prospective study.

## 1. Introduction

Atrial fibrillation (AF) is the most sustained arrhythmia in the clinical setting. AF increases the risk of atrial thrombus, most commonly in the left atrial appendage (LAA) (>90%) [1]. Transesophageal echocardiography (TEE) was performed before catheter ablation or percutaneous LAA closure to exclude the left atrium (LA) or LAA thrombus (LAAT). Oral anticoagulation (OAC) therapy was recommended in patients with LAAT. Vitamin K antagonists (VKAs), such as warfarin, were commonly used, with the therapeutic international normalized ratio (INR) of 2.0 to 3.0. In the past decade, non-vitamin K antagonist oral anticoagulants (NOACs) have been widely used for thromboembolic prevention. Standard-dose NOACs were recommended in the guidelines. However, low-dose NOACs were suggested in some special subset of patients, such as patients aged ≥75 years, weighted <50 kg, or with creatinine clearance (CrCl) <50 mL/min [2]. Low-dose NOACs in Asian population showed noninferior safety and efficacy in stroke prevention compared with standard-dose NOACs [3, 4]. Previous investigations indicated that standard-dose NOACs were effective in LAAT resolution [5, 6]. Ke et al. [5] compared the efficacy and safety on the resolution of LA/LAA thrombus between rivaroxaban and warfarin. They found that rivaroxaban 20 mg was more effective than warfarin on the resolution of LA/LAA thrombus in nonvalvular AF patients especially after 6-week treatments. Lin et al. [6] found that both dabigatran and rivaroxaban (81.8% vs. 83.3% complete resolution) are potential options for treating LA/LAA thrombus in patients with nonvalvular AF. However, the safety and efficacy for the treatment of LAAT by low-dose NOACs compared to standard-dose NOACs were still unknown. In this study, we aimed to evaluate the safety and efficacy of standard- and low-dose NOACs in the resolution of LAAT in patients with nonvalvular AF.

## 2. Methods

### 2.1. Study Population

Nonvalvular AF patients who were scheduled to undergo catheter ablation or percutaneous LAA closure in Ningbo First Hospital between January 2014 and September 2019 were retrospectively screened. The inclusion criteria were as follows: (1) nonvalvular AF with LAAT confirmed by TEE; (2) treated with NOACs; (3) underwent repeated TEE. The exclusion criteria were as follows: (1) patients with mechanical valves or moderate-to-severe mitral stenosis; (2) treated with warfarin; (3) absence of repeated TEE; (4) uncontrolled bleeding diseases; (5) CrCl <30 mL/min. The demographic and clinical data were collected, including age, gender, and comorbidities. CHA_2_DS_2_-VASc and HAS-BLED scores were calculated [7, 8]. Serum creatinine was recorded, and CrCl was calculated by the Cockcroft–Gault equation [9].

This study was conducted in compliance with the law-protecting personal data in accordance with the guidelines of the Helsinki Declaration. The study was approved by the Ethics Committee of Ningbo First Hospital.

### 2.2. Initial and Follow-Up

TEE was performed using a Philips EPIQ 7C device (Philips, Amsterdam, Netherlands). The gain was continuously adjusted until acquisition of the best image. The presence or absence of LAAT was determined by 2 experienced echocardiographers. LAAT was defined as well-circumscribed, highly reflective mass with texture different from that of the atrial wall and with uniform consistency [10]. The first follow-up TEE was arranged 1 month from the initial TEE. If the LAAT was not completely resolved, repeated TEE was performed 1 month later. The thrombus outcome criteria were defined as follows: resolved = if no thrombus was detectable on the follow-up TEE; reduced = if the thrombus was smaller than at baseline (change >1 mm); unchanged = if the change was <1 mm.

### 2.3. Strategy for NOACs' Dose Choice

Low-dose NOACs were used in patients aged ≥75 years, weighted <50 kg, or with creatinine clearance (CrCl) <50 mL/min: dabigatran 110 mg, twice daily; rivaroxaban 15 mg, once daily. The other patients were recommended to take standard-dose NOACs: dabigatran 150 mg, twice daily; rivaroxaban 20 mg, once daily.

### 2.4. Clinical Outcomes

Clinical outcomes included death, ischemic stroke, transient ischemic attack (TIA), systemic embolism, and bleeding events. Stroke was defined as the onset of a new neurologic deficit that occurred any time after LAAC and persisted for >24 hours. It was confirmed by cerebral magnetic resonance imaging or CT and determined by at least two radiologists or neurologists. If the duration of the deficit was <24 hours, it was defined as a TIA. Bleeding events were classified as major (intracranial, retroperitoneal, intraspinal, intraocular, or pericardial hemorrhage; decrease in hemoglobin >2 g/dL; transfusion of ≥2 units of packed red blood cells) or minor (remaining types of bleeding events) 11.

### 2.5. Statistical Analysis

Based on the dose of NOACs, patients were divided into 2 groups: standard-dose group and low-dose group. Normally distributed continuous variables were expressed as the mean (standard deviation), while the median (interquartile range) was used for variables with a skewed distribution. Categorical variables were expressed as absolute numbers (percentages). Continuous variables were compared using the *t*-test and Mann–Whitney *U* test for normally and nonnormally distributed data, respectively. Categorical variables were compared using the chi-square test or Fisher's exact test where appropriate. A value of *P* <0.05 was considered as statistical significance. All analyses were performed using SPSS 19.0 (IBM, Armonk, NY, USA).

## 3. Results

### 3.1. Baseline Characteristics

A total of 24 nonvalvular AF patients with LAAT and who took NOACs were included. Standard-dose NOACs were used in 14 patients, while low-dose NOACs were used in 10 patients (4 aged ≥75 years, 2 weighted <50 kg, and 4 with CrCl <50 mL/min) (Figure 1). Patients in the low-dose group were older than those in the standard-dose group. The CHA_2_DS_2_-VASc and HAS-BLED scores were higher in the low-dose group. The percentages of hypertension, congestive heart failure, and previous stroke/TIA were higher in the low-dose group. The level of CrCl was significantly lower in the low-dose group. The mean values of LA diameter, LVEF, and LAA orifice diameter were comparable between groups (Table 1).

### 3.2. Resolution of LAAT

The resolution of LAAT is shown in Table 2. In the standard-dose group, repeated TEE indicated that LAAT in 4 patients was completely resolved, 8 reduced, and 2 unchanged after 1 month. In the remaining 10 patients, LAAT in 4 patients was completely resolved, 4 reduced, and 2 unchanged 1 month later. In the remaining 6 patients, LAAT in 4 patients was completely resolved, 1 reduced, and 1 unchanged 1 month later. In the low-dose group, repeated TEE indicated that LAAT in 3 patients was completely resolved, 5 reduced, and 2 unchanged after 1 month. In the remaining 7 patients, LAAT in 3 patients was completely resolved, 3 reduced, and 1 unchanged 1 month later. In the remaining 4 patients, LAAT in 2 patients was completely resolved and 2 unchanged 1 month later. Totally, LAAT in 85.7% (12/14) and 80% (8/10) of patients was completely resolved in the standard-dose group and low-dose group, respectively. The percentage of completely resolved was comparable between the two groups.

### 3.3. Clinical Outcomes

No death, TIA/stroke, systemic embolism, or major bleeding event occurred during the treatment of LAAT in the two groups. One patient in the standard-dose group had slight hemorrhinia, while 1 in the low-dose group experienced gingival bleeding. Both patients neither discontinued NOACs nor adjusted the dose.

## 4. Discussion

In the present study, some special patients with LAAT received low-dose NOACs according to the guideline. Complete LAAT resolution was comparable between the two groups. No major adverse events occurred during the treatment of LAAT.

The majority of thrombi was originated from LAA in nonvalvular AF patients [1]. Warfarin was recommended to prevent thromboembolic events. However, the impact of food and drugs on warfarin requires frequent monitoring of INR and dose adjustment, making it difficult for many patients to use warfarin in the clinical setting [12]. The NOACs work by direct inhibition of either thrombin (e.g., dabigatran) or factor Xa (e.g., rivaroxaban) to prevent thrombus formation. Many clinical trials have compared NOACs and warfarin in nonvalvular AF patients [13, 14]. NOACs offer several lifestyle and therapeutic advantages for patients relative to warfarin. Therefore, these alternative agents are increasingly used in the thromboembolic prevention [15].

Previous studies showed that both dabigatran and rivaroxaban are potential therapeutic options for resolution of LAAT. Ke et al. [5] conducted a randomized controlled trial of rivaroxaban versus warfarin for LA thrombus in 80 subjects. Complete resolution was observed in 6 patients treated with rivaroxaban while none in those with warfarin at 6 weeks (*P* = 0.011). Another follow-up TEE was performed at 12 weeks, with complete resolution observed in 32 (80%) and 28 (70%) subjects in the rivaroxaban group and warfarin group, respectively (*P* = 0.302). Lin et al. 6 included 34 patients with LA/LAAT and treated with NOACs (12 dabigatran and 22 rivaroxaban). Finally, thrombus resolution was achieved in 83.3% and 81.8% of patients treated with dabigatran and rivaroxaban, respectively. Some other studies also confirmed the efficacy of NOACs in the treatment of LAAT [16–18]. However, standard-dose NOACs were commonly used in those investigations.

The dose of NOACs in Asian population was still controversial. The bleeding risk was higher in Asian population when taking OACs [19]. Therefore, many physicians may prescribe low-dose NOACs to nonvalvular AF patients. In the nationwide retrospective cohort study collected from Taiwan National Health Insurance Research Database, only 12% and 6% of patients took standard-dose dabigatran (150 mg, twice daily) and rivaroxaban (20 mg, once daily), respectively [20]. J-ROCKET AF trial revealed that low-dose rivaroxaban (15 mg, once daily) was comparable with warfarin in thromboembolic prevention in Japanese population [21]. In a Korean investigation, both standard- and low-dose dabigatran showed similar efficacy in stroke prevention with warfarin. However, low-dose dabigatran reduced the major bleeding risk [4]. Previous studies have proved the efficacy and safety of low-dose NOACs in AF patients for stroke prevention, whereas no data regarding the efficacy and safety of low-dose NOACs in the treatment of LAAT have been published. The present study included patients with LAAT treated with both standard-dose and low-dose NOACs. According to the guidelines, low-dose NOACs were prescribed to some special patients. We found that the percentages of complete resolution were both high and comparable between the low-dose group and standard-dose group.

The present study has several limitations. It was a single-center, retrospective study with a relatively small number of samples. More comprehensive investigation is needed with a larger study cohort in the future. Finally, low-dose NOACs were only used in some special subset of patients. Whether the results can be extended to the whole nonvalvular AF population is known.

## 5. Conclusion

Low-dose NOACs are a safe and effective option for the treatment of LAAT in some special subset patients. However, the results warrant validation in a prospective study.

## Figures and Tables

**Figure 1:** The distribution of dabigatran and rivaroxaban usage in the standard-dose and low-dose groups. The doses of NOACs for patients in the standard-dose group were dabigatran 150 mg (twice daily) and rivaroxaban 20 mg (once daily), while those for patients in the low-dose group were dabigatran 110 mg (twice daily) and rivaroxaban 15 mg (once daily).

**Table 1:** Baseline characteristics.

	Standard-dose group	Low-dose group	*P* value
*n*	14	10	—
Age, years	64.4 ± 5.9	68.9 ± 9.6	0.171
Male, *n* (%)	7 (50)	5 (50)	1.000
Persistent AF, *n* (%)	5 (35.7)	4 (40)	1.000
Hypertension, *n* (%)	8 (57.1)	8 (80)	0.388
Diabetes mellitus, *n* (%)	3 (21.4)	2 (20)	1.000
Congestive heart failure, *n* (%)	2 (14.3)	2 (20)	1.000
Previous TIA/stroke, *n* (%)	4 (28.6)	4 (40)	0.673
Previous bleeding, *n* (%)	3 (21.4)	2 (20)	1.000
CHA_2_DS_2_-VASc score, points	3 (2.5, 4)	4 (3, 6)	0.049
HAS-BLED score, points	1.5 (1, 2)	2.5 (2, 4)	0.069
CrCl, mL/min	96.4 ± 10.1	68.5 ± 9.6	<0.001
LA diameter, mm	44.2 ± 8.6	45.3 ± 5.8	0.731
LVEF, %	57.0 ± 12.8	58.6 ± 12.1	0.760
LAA orifice diameter, mm	21.0 ± 3.0	21.8 ± 2.8	0.521

AF: atrial fibrillation; TIA: transient ischemic attack; CrCl: creatinine clearance; LA: left atrium; LVEF: left ventricular ejection fraction; LAA: left atrial appendage.

**Table 2:** LAAT resolution by different doses of NOACs.

	Standard-dose group (*n* = 14)			Low-dose group (*n* = 10)		
	Resolved	Reduced	Unchanged	Resolved	Reduced	Unchanged
1 month	4	8	2	3	5	2
2 months	4	4	2	3	3	1
3 months	4	1	1	2	0	2
Total, *n* (%)	12 (85.7)	1 (7.1)	1 (7.1)	8 (80)	1 (10)	1 (10)

## Data Availability

The data used to support the findings of this study are available from the corresponding author upon request.

## References

[1] Al-Saady N. M., Obel O. A., Camm A. J. (1999). Left atrial appendage: structure, function, and role in thromboembolism. *Heart*.

[2] Hindricks G., Potpara T., Dagres N. (2021). 2020 ESC Guidelines for the diagnosis and management of atrial fibrillation developed in collaboration with the European Association for Cardio-Thoracic Surgery (EACTS). *European Heart Journal*.

[3] Hori M., Matsumoto M., Tanahashi N. (2014). Rivaroxaban vs. warfarin in Japanese patients with non-valvular atrial fibrillation in relation to age. *Circulation Journal*.

[4] Lee K. H., Park H. W., Lee N. (2017). Optimal dose of dabigatran for the prevention of thromboembolism with minimal bleeding risk in Korean patients with atrial fibrillation. *Europace*.

[5] Ke H. H., He Y., Lv X. W., Zhang E. H, Wei Z., Li J. Y. (2019). Efficacy and safety of rivaroxaban on the resolution of left atrial/left atrial appendage thrombus in nonvalvular atrial fibrillation patients. *Journal of Thrombosis and Thrombolysis*.

[6] Lin C., Quan J., Bao Y., Xie Y., Wei Y., Ling T., Pan W., Wu L., Xie Y. (2020). Outcome of non-vitamin K oral anticoagulants in the treatment of left atrial/left atrial appendage thrombus in patients with nonvalvular atrial fibrillation. *Journal of Cardiovascular Electrophysiology*.

[7] Lip G. Y., Nieuwlaat R., Pisters R., Lane D. A., Crijns H. J. (2010). Refining clinical risk stratification for predicting stroke and thromboembolism in atrial fibrillation using a novel risk factor-based approach: the euro heart survey on atrial fibrillation. *Chest*.

[8] Pisters R., Lane D. A., Nieuwlaat R., De Vos C. B., Crijns H. J., Lip G. Y. (2010). A novel user-friendly score (HAS-BLED) to assess 1-year risk of major bleeding in patients with atrial fibrillation: the Euro Heart Survey. *Chest*.

[9] Cockcroft D. W., Gault M. H. (1976). Prediction of creatinine clearance from serum creatinine. *Nephron*.

[10] Hahn R. T., Abraham T., Adams M. S. (2013). Guidelines for performing a comprehensive transesophageal examination: recommendations from the American society of echocardiography and the society of cardiovascular anesthesiologist. *Journal of the American Society of Echocardiography*.

[11] Schulman S., Kearon C. (2005). Definition of major bleeding in clinical investigations of antihemostatic medicinal products in non-surgical patients. *Journal of Thrombosis and Haemostasis*.

[12] Go A. S., Hylek E. M., Borowsky L. H., Phillips K. A., Selby J. V., Singer D. E. (1999). Warfarin use among ambulatory patients with nonvalvular atrial fibrillation: the anticoagulation and risk factors in atrial fibrillation (ATRIA) study. *Annals of Internal Medicine*.

[13] Connolly S. J., Ezekowitz M. D., Yusuf S. (2009). Dabigatran versus warfarin in patients with atrial fibrillation. *New England Journal of Medicine*.

[14] Patel M. R., Mahaffey K. W., Garg J. (2011). Rivaroxaban versus warfarin in nonvalvular atrial fibrillation. *New England Journal of Medicine*.

[15] Hale Z. D., Kong X., Haymart B. (2017). Prescribing trends of atrial fibrillation patients who switched from warfarin to a direct oral anticoagulant. *Journal of Thrombosis and Thrombolysis*.

[16] Fleddermann A., Eckert R., Muskala P., Hayes C., Magalski A., Main M. L. (2019). Efficacy of direct acting oral anticoagulant drugs in treatment of left atrial appendage thrombus in patients with atrial fibrillation. *The American Journal of Cardiology*.

[17] Hussain A., Katz W. E., Genuardi M. V. (2019). Non-vitamin K oral anticoagulants versus warfarin for left atrial appendage thrombus resolution in nonvalvular atrial fibrillation or flutter. *Pacing and Clinical Electrophysiology*.

[18] Murtaza G., Turagam M. K., Atti V. (2020). Warfarin vs non-vitamin K oral anticoagulants for left atrial appendage thrombus: a meta-analysis. *Journal of Cardiovascular Electrophysiology*.

[19] Chao T. F., Chen S. A., Ruff C. T. (2019). Clinical outcomes, edoxaban concentration, and anti-factor Xa activity of Asian patients with atrial fibrillation compared with non-Asians in the ENGAGE AF-TIMI 48 trial. *European Heart Journal*.

[20] Chan Y. H., See L. C., Tu H. T. (2018). Efficacy and safety of apixaban, dabigatran, rivaroxaban, and warfarin in asians with nonvalvular atrial fibrillation. *J Am Heart Assoc*.

[21] Hori M., Matsumoto M., Tanahashi N. (2012). Rivaroxaban vs. warfarin in Japanese patients with atrial fibrillation - the J-ROCKET AF study. *Circulation Journal*.

